The article "The Importance of Early Identification for Parkinson's Disease Patients with Postural Instability and Gait Disturbance" was retracted in 2023. Reasons: signs of a paper mill; compromised peer review; unreliable results or conclusions.

# The Importance of Early Identification for Parkinson's Disease Patients with Postural Instability and Gait Disturbance

**DOI:** 10.1155/2022/6701519

**Published:** 2022-11-18

**Authors:** You Wu, Yi-Wen Yang, Si-Chun Gu, Yu Zhang, Rong Shi, Chang-De Wang, Can-Xing Yuan, Qing Ye

**Affiliations:** ^1^Department of Neurology, Longhua Hospital, Shanghai University of Traditional Chinese Medicine, 725 South Wanping Road, Shanghai 200032, China; ^2^School of Chinese Materia Medica, Shanghai University of Traditional Chinese Medicine, 1200 Cailun Road, Pudong New District, Shanghai 201203, China; ^3^Department of Neurology, Xinhua Hospital, Shanghai Jiao Tong University School of Medicine, 665 Kongjiang Road, Shanghai 200092, China; ^4^Department of Emergency, Shuguang Hospital, Shanghai University of Traditional Chinese Medicine, 528 Zhangheng Road, Shanghai 201203, China; ^5^Department of Neurology, Shanghai TCM-integrated Hospital, Shanghai University of Traditional Chinese Medicine, 230 Baoding Road, Shanghai 200082, China

## Abstract

**Background:**

More and more evidence-based medicine has proved that Parkinson's disease (PD) patients of tremor-dominant (TD) and postural instability and gait difficulty (PIGD) subtype express great individual differences and heterogeneity. Early identification of different subtypes may be an important way to delay disease progression and improve patients' prognosis.

**Objective:**

The study aimed to compare the spectrum of motor symptoms (MS) and nonmotor symptoms (NMS) between TD and PIGD dominant in the early and middle stages of PD, and determine predictive factors that are associated with different motor subtypes.

**Methods:**

292 PD patients in this study were divided into TD-PD and PIGD-PD, and the clinical characteristics between different motor subtypes were compared based on scales related to sleep, mood, and autonomic function. Univariate and multivariate ordered logistic regression analyses were used to analyze the independent influencing factors of disease severity between different motor subtypes. Through the establishment of binary logistic regression model, the potential independent risk factors for distinguishing TD-PD and PIGD-PD were studied.

**Results:**

Compared with TD subtype, patients with PIGD subtype have longer course of disease, higher disease severity, and higher daily dosage of levodopa. The severity of nontremor motor symptoms in PIGD-PD is greater than that of TD subtype. Only PIGD score was independently associated with disease severity for the two motor subtypes. Meanwhile, high scores (LED, total UPDRS, PIGD score, gastrointestinal, thermoregulatory, RBDSQ) and low tremor scores were the potential independent risk factors for distinguishing PIGD-PD from TD-PD.

The article "The Importance of Early Identification for Parkinson's Disease Patients with Postural Instability and Gait Disturbance" was retracted in 2023. Reasons: signs of a paper mill; compromised peer review; unreliable results or conclusions.

**Conclusion:**

Specific nonmotor symptoms (RBD, gastrointestinal function and thermoregulation function) were associated with the PIGD subtype. Prompt detection and early treatment of NMSs related to the PIGD subtype based on the treatment of motor symptoms may improve patient outcomes.

## 1. Introduction

Parkinson's disease (PD) is a common chronic, progressive, and degenerative disease of the nervous system. More and more evidence-based medicine has proved that the clinical manifestations of PD are complex and diverse, including tremor, rigidity, bradykinesia, postural instability, etc. [1]. These symptoms are important factors that affect the quality of life of PD patients and even bring progressive functional disability [2]. Moreover, due to the different factors of patients' constitution, genetics, and so on, their clinical symptoms, onset age, and progress rate express great individual differences and heterogeneity [3]. The study of the clinical characteristics of the PD patients is helpful to further understand the pathogenesis, clinical progress, and individualized treatment of PD.

To reflect the clinical heterogeneity of PD objectively, scholars have analyzed PD patients utilizing data-driven classification technology. One of the most common groupings is tremor-dominant (TD) versus postural instability and gait difficulty (PIGD) subtypes [4, 5]. After comparing the clinical characteristics of TD and PIGD patients, it was uncovered that most PD patients of PIGD subtype have rapid disease progression and poor clinical prognosis [6]. This kind of clinical heterogeneity may reflect the potential biological or pathophysiological differences between patients; however, the origin and mechanism of the two subtypes remain unclear.

In addition to typical motor symptoms, many of the PD patients are accompanied by some nonmotor symptoms like sleep disorder, depression and anxiety, hyposmia, and gastrointestinal disorder which often exist before the diagnosis of PD and may be a critical precursor feature of PD [7]. The NMS may differ between TD and PIGD subtypes, as well as their severity and prognosis. Some clinical reports suggest that patients of PIGD subtype have a higher risk of cognitive impairment, dementia, and hallucinations, as well as psychological and emotional problems such as depression and indifference, and these symptoms usually have no or poor response to dopaminergic therapy. In contrast, TD subtype is characterized by milder clinical symptoms, slower progression of motor and cognitive symptoms, and a lower risk of dementia and mental illness [8].

The article "The Importance of Early Identification for Parkinson's Disease Patients with Postural Instability and Gait Disturbance" was retracted in 2023. Reasons: signs of a paper mill; compromised peer review; unreliable results or conclusions.

Thus, on the basis of the treatment of motor symptoms, early identification of different subtypes and individualized intervention of the nonmotor symptoms related to the subtypes may be an important way to delay disease progression and improve patients' prognosis. However, most of the previous studies were based on a single nonmotor symptom questionnaire, and few studies were reported on distinguishing the nonmotor symptoms of different subtypes. To address these gaps in knowledge, our team carried out a cross-sectional study in a multi-center cohort of early and middle-stage PD in China, aiming to analyze the independent influencing factors between the two different motor subtypes.

## 2. Patients and Methods

### 2.1. Study Population

In this multi-center cross-sectional study, PD patients were recruited from Parkinson's disease clinic of 4 university hospitals in Shanghai (Longhua Hospital Affiliated to Shanghai University of TCM, Xinhua Hospital Affiliated to Shanghai Jiao Tong University School of Medicine, Shanghai TCM-integrated Hospital Affiliated to Shanghai University of TCM, and Shuguang Hospital Affiliated to Shanghai University of TCM) from December 2015 to December 2018.

Inclusion criteria are as follows: ① aged between 30 and 80; ② diagnosed as idiopathic PD according to the Movement Disorder Society (MDS) Clinical Diagnostic Criteria; and ③ the Hoehn and Yahr stages 1–3 [9, 10].

Exclusion criteria are as follows: ① receiving treatments for psychiatric disorders; ② secondary PD; ③ with other serious central nervous system diseases; ④ with severe heart, lung, kidney disease, and mental illness; ⑤ drug or alcohol abuse; and ⑥ pregnant or lactating.

This study was approved by the Ethics Committee of Longhua Hospital. Demographic characteristics and clinical features, including gender, age, age of onset, disease duration, individual anti-PD drugs, and dosage, were collected for all study participants. The studies involving human participants were reviewed and approved by the Ethics Committee of Longhua Hospital with the following ethic code: 2017LCSY326. All participants gave their informed consent for inclusion before they participated in the study (trial registration: Chinese Clinical Trial Register, ChiCTR-INR-17011949).

### 2.2. Subtype Classifications

The motor subtype in our study was divided by the Unified Parkinson's Disease Rating Scale (UPDRS) following the method proposed by Jankovic et al. The ratio of the mean tremor score (the average of UPDRS III items 20-21 and UPDRS II item 16) and the mean PIGD score (the average of UPDRS III items 29 and 30 and UPDRS II items 13–15) was used to determine the motor subtypes. When the ratio was ≥1.5, ≤1.0, or between 1.0 and 1.5, the patients were defined as TD, PIGD, and mixed subtypes, respectively [4]. Twenty-two participants classified as “mixed subtype” were not excluded in the further analysis. In our study, there were 148 patients in the TD subtype and 122 patients in the PIGD subtype.

The article "The Importance of Early Identification for Parkinson's Disease Patients with Postural Instability and Gait Disturbance" was retracted in 2023. Reasons: signs of a paper mill; compromised peer review; unreliable results or conclusions.

### 2.3. Collection of Clinical Data

The following scales were used to assess all participants face-to-face by well-trained movement disorder neurologists.

The Unified Parkinson's Disease Rating Scale (UPDRS; Part I: mentation, behavior, and mood; Part II: activities of daily living; Part III: motor examination; Part IV: treatment complications) was used for general assessment of PD severity. In the UPDRS Part II and III, we subdivided motor disability into four subscores, including tremor score (items 16, 20, 21), rigidity score (item 22), bradykinesia score (items 23-26, 31), PIGD score (items 13-15, 29, 30).

Autonomic symptoms were investigated using the Scales for Outcomes in Parkinson's Disease–Autonomic Dysfunction (SCOPA-AUT). The SCOPA-AUT assesses the following regions: gastrointestinal (Q1-7), urinary (Q8-13), cardiovascular (Q14-16), thermoregulatory (Q17-21), pupillomotor (Q19), and sexual dysfunction (Q22-25). The SCOPA-AUT total score ranges from 0 to 69, with higher scores reflecting worse autonomic functioning.

RBDSQ contains 13 questions, covering several aspects of RBD symptom spectrum, and a score greater than or equal to 5 is used as the cut-off value for possible RBD [11]. We used the Parkinson's Disease Sleep Scale (PDSS) to examine the sleep disturbances and nocturnal problems of PD patients. Each item score ranges from 0 to 10, and lower score indicates more severe symptom. We used Hamilton Depression Rating Scale (HAMD) to screen for PD depression and Hamilton Anxiety Rating Scale (HAMA) to assess the severity of anxiety symptoms. The HAMA is grouped into two subscales for measuring the psychic anxiety (items 1-6 and 14) and somatic anxiety (items 7–13), respectively.

### 2.4. Statistical Analysis

Descriptive statistics were conducted for the demographic characteristics and PD clinical scales of our study group according to data characteristics. All continuous variables were tested for normality using Kolmogorov–Smirnov test and were expressed as mean ± standard deviation or median (interquartile range). Categorical variables were described as number (percentage). The comparisons between the TD-PD and PIGD-PD were performed by using Student's *t* tests or Mann–Whitney *U* tests for continuous variables, while chi-square tests or Fisher's exact tests for categorical variables. The prevalence of each nonmotor symptom between two different PD motor subtypes was analyzed using chi-square test. We used univariate and multivariate ordered logistic regression analyses to evaluate the correlation between PD clinical symptoms and disease severity of different motor subtypes. A binary logistic regression model was performed to explore the potential independent risk factors in differentiating between the TD-PD and PIGD-PD. Setting TD and PIGD subtype as the dependent variable, respectively, significant candidate factors having *P* < 0.05 at univariate analysis were entered in the multivariate analysis as independent covariables. Contribution of each factor was presented as beta coefficients and odds ratios (ORs) with 95% confidence intervals (95% CIs). Receiver operating characteristic (ROC) curves were created through the binary logistic regression model. Areas under the curve (AUC) of the ROC curves were utilized to evaluate the accuracy of the model, and the maximum value of the Youden index (sensitivity + specificity−1) was calculated to acquire the cut-off values of each risk factor. All statistical analyses were performed by SPSS version 25.0 for Windows (IBM Corp., Armonk, NY). The level of statistically significance was predefined as *P* < 0.05 (two-sided).

The article "The Importance of Early Identification for Parkinson's Disease Patients with Postural Instability and Gait Disturbance" was retracted in 2023. Reasons: signs of a paper mill; compromised peer review; unreliable results or conclusions.

## 3. Results

### 3.1. Demographic and Clinical Characteristics of Participants

Among the included 292 patients (66.7 ± 9.0 years old, 55.1% males), 148 (50.7%) patients were classified as the TD subtype and 122 (41.8%) were grouped with the PIGD subtype. Of the whole group, the average age of disease onset was 61.6 ± 9.9 years and the mean disease duration was 5.2 ± 4.2 years. The majority of the patients were in the early stage of the disease with an average Hoehn and Yahr stage of 1.8 ± 0.6 (77.4% stage I–II). There was no significant difference between the two subtypes in terms of gender, age, education, PD family history, and age of onset. However, compared to the TD-PD, PIGD-PD had longer disease duration (*P*=0.001), more advanced Hoehn and Yahr stage (*P* < 0.001), and higher daily levodopa equivalent dose (*P* < 0.001; Table 1).

The clinical characteristics of TD-PD and PIGD-PD patients are summarized in Table 2. As can be seen from the Unified Parkinson's Disease Rating Scale, all parts of UPDRS in PIGD-PD patients were more severe than TD-PD patients, except UPDRS IV. Meanwhile, we observed significantly higher PIGD, bradykinesia scores in PIGD-PD, while higher tremor score in TD-PD. There was no significant difference in rigidity score between TD-PD and PIGD-PD. In terms of nonmotor symptoms, PIGD-PD had higher RBDSQ, SCOPA-AUT, HAMA, and HAMD scores, especially in gastrointestinal, thermoregulatory, and somatic anxiety symptoms. Furthermore, there was no significant difference between the two different motor subtypes on the PDSS.

The article "The Importance of Early Identification for Parkinson's Disease Patients with Postural Instability and Gait Disturbance" was retracted in 2023. Reasons: signs of a paper mill; compromised peer review; unreliable results or conclusions.

### 3.2. Prevalence of Nonmotor Symptoms of PD Patients between Different Motor Subtypes

Differences in the prevalence of NMS among different motor subtypes were observed, with PIGD-PD patients reporting significantly more gastrointestinal, thermoregulatory, anxiety, and depression symptoms compared to TD-PD patients, particularly in dysphagia (32.8% vs 9.5%, respectively, *P* < 0.001), constipation (74.6% vs 49.3%, respectively, *P* < 0.001), RBD (31.1% vs 11.5%, respectively, *P* < 0.001), and depression (97.5% vs 75.7%, respectively, *P* < 0.001) (Table 3).

### 3.3. Influence Factors of Disease Severity between Different Motor Subtypes

As can be seen from Figure 1, the proportion of TD-PD patients with early stage of Parkinson's disease (H&Y stage <2.0) accounted for 64.1%, while PIGD-PD accounted for 34.5%. On the contrary, PIGD-PD had a larger proportion of patients with middle stage of PD (H&Y stage 2.0-3.0) compared to TD-PD subtype (65.5% vs 35.9%, *P* < 0.001). Obviously, the disease severity of PIGD-PD is greater than that of TD-PD. We further performed univariable and multivariable logistic regression analyses to identify the influence factors of disease severity in patients with different motor subtypes, as presented in Table 4. Among the four motor subscores, in Table 5PIGD score (TD-PD (OR 1.207, 95% CI 0.882–1.652, *P*=0.039); PIGD-PD (OR 1.922, 95% CI 1.438–2.568, *P* < 0.001)) was independently associated with disease severity for the two motor subtypes. Moreover, we found higher disease duration (OR 1.332, 95% CI 1.194–1.486, *P* < 0.001) and LED (mg/day) (OR 1.002, 95% CI 1.000–1.004, *P*=0.011) was associated with disease severity of TD-PD patients, whereas higher gastrointestinal scores (OR 1.406, 95% CI 1.073–1.841, *P*=0.036) correlated with disease severity of PIGD-PD (Tables 4 and 5).

### 3.4. Independent Risk Factors of Different Motor Subtypes

The abovementioned results indicated the profound impact of PIGD score on disease severity, and PIGD-PD patients performed more serious symptoms. In a further step, in order to differentiate PIGD-PD from TD-PD, we performed binary logistic regression analysis to identify the independent risk factors for different motor subtypes. The logistic regression model correctly classified 85.4% of cases. The following factors were found to be positive correlation with risk of PIGD-PD, after eliminating potential interference by confounding factors (Table 6): LED (OR 1.004, 95% CI 1.001–1.007; *P*=0.022); total UPDRS (OR 1.198, 95% CI 1.014–1.416; *P*=0.034); PIGD score (OR 4.116, 95% CI 1.981–8.552; *P* < 0.001); gastrointestinal (OR 1.808, 95% CI 0.916–3.569; *P*=0.048); thermoregulatory (OR 1.974, 95% CI 0.932–4.182; *P*=0.046); RBDSQ (OR 1.416, 95% CI 1.053–1.903; *P*=0.021). Only the tremor score (OR 68.126, 95% CI 15.124–306.862; *P* < 0.001) was the independent risk factor for TD-PD (Table 7).

The article "The Importance of Early Identification for Parkinson's Disease Patients with Postural Instability and Gait Disturbance" was retracted in 2023. Reasons: signs of a paper mill; compromised peer review; unreliable results or conclusions.

ROC curve analyses were performed to evaluate the model and to ascertain the optimum cut-off value of the above risk factors: levodopa equivalent dose of more than 331 mg per day (*P* < 0.001, AUC 0.681), total UPDRS = 26.5 (*P* < 0.001, AUC 0.662), PIGD score = 3.5 (*P* < 0.001, AUC 0.802), gastrointestinal score = 4.5 (*P* < 0.001, AUC 0.743), thermoregulatory score = 1.5(*P* < 0.001, AUC 0.665), RBDSQ score = 2.5 (*P* < 0.001, AUC 0.702), and tremor score (*P* < 0.001, AUC 0.892). These factors discriminated PIGD-PD from TD-PD (Table 8, Figure 2).

## 4. Discussion

### 4.1. PIGD-PD Has Higher Disease Severity

In the 1980s, Zetusky et al. first discovered the heterogeneity of PD in motor symptoms. PD patients with tremor had fewer dysfunction than those with other movement symptoms [12]. In 1990, PD is further divided into TD subtype and PIGD subtype according to the characteristics of motor symptoms. Thereafter, relevant scholars have carried out clinical studies on different subtypes of PD [4]. We compared the clinical features of 270 patients with TD-PD and PIGD-PD, including the evaluation of MS and NMS score. It turned out that PIGD-PD has higher disease severity as expected.

In terms of the MS score, PIGD-PD has more severe axial symptoms such as postural instability, gait disorder, and bradykinesia and the motor symptoms of TD-PD are relatively milder. Meanwhile, for the severity and incidence of NMS in different motor subtypes, several studies compared the autonomic nervous function of TD subtype and PIGD subtype with NMS Quest scale [13–15]. In this study, a more comprehensive NMS evaluation scale has been taken and it was uncovered that PIGD-PD generally has higher severity and incidence of NMS, especially in gastrointestinal symptoms, thermoregulation, RBD, anxiety, and depression.

The neuropathological manifestations may account for a different severity and incidence of NMS between the two subtypes. Many studies have found that the decrease of dopamine neurons in substantia nigra of PIGD-PD is more serious than that of TD-PD [16–18]. The higher disease severity of PIGD-PD may be attributed to more dopamine consumption in striatum. These more severe motor and nonmotor symptoms may directly affect the survival time and quality of life of PIGD-PD.

### 4.2. The Gastrointestinal Dysfunction, RBD, and Thermoregulation Disorder Are Independent Risk Factors for PD

We further analyzed the influencing factors of disease severity in TD-PD and PIGD-PD, which found that PIGD score is an independent influencing factor shared by the two subtypes. PIGD score is also one of the key indicators to distinguish between TD-PD and PIGD-PD. Due to the differences in disease severity and progression between the two subtypes, early identification and intervention of TD-PD and PIGD-PD are very necessary.

The article "The Importance of Early Identification for Parkinson's Disease Patients with Postural Instability and Gait Disturbance" was retracted in 2023. Reasons: signs of a paper mill; compromised peer review; unreliable results or conclusions.

Clinically, PD patients are usually diagnosed in stage 3∼4 of Braak stage. At this time, typical motor symptoms of tremor, rigidity, and hypokinesia have already appeared. However, autonomic nerve dysfunction, such as gastrointestinal, parasomnias, mood changes, and other NMS, may have existed several years before the emergence of typical motor symptoms, corresponding to stage 1∼2 of Braak stage [19].

Therefore, according to the performance difference between TD and PIGD in NMS, this study determined the influencing factors of different motor subtypes in NMS through binary logistic regression. We found that gastrointestinal dysfunction, RBD, and thermoregulation disorder are positively correlated with PIGD, but vice versa in TD type.

The results of investigations on the relationship between NMS and PD displayed that 80% of rapid eye movement sleep behavior disorder (RBD) patients will progress to PD within 10–12 years [20–22]; 67.5% of PD patients have one or more gastrointestinal symptoms before the onset of motor symptoms, and constipation is a typical PD precursor biomarker [13]; in comparison with PD patients without hyperhidrosis, those with hyperhidrosis have higher dyskinesia scores [23, 24]. In addition, some clinical reports have found that the treatment of RBD and gastrointestinal symptoms, such as low-dose clonazepam and defecation drugs, also contributes to the improvement of Parkinson's symptoms [25, 26].

It can be seen that while treating MS, the early identification of TD-PD and PIGD-PD and the intervention for RBD, gastrointestinal symptoms, and thermoregulation disorders may further improve the life quality of patients and delay the progress of the disease.

### 4.3. Regulating Circadian Disruption May Be Another Approach for Early Intervention in PIGD-PD Patients

This study found that RBD, gastrointestinal symptoms, and thermoregulation disorders were correlated with PIGD-PD. It can be seen that the three are not completely independent, but have some relationship. It was speculated that this relationship may be related to circadian rhythm disturbances.

In recent years, studies on neurodegenerative diseases proved that circadian rhythm disturbances are prevalent in neurodegenerative diseases and may be the precursor of the occurrence and progression of neurodegenerative diseases. Data from related studies on PD and circadian rhythm disturbances uncovered that circadian rhythm disturbances can be manifested as oxidative stress, causing neuroinflammatory response, and the damage of dopamine neurons can accelerate the progression of PD [27]. Meanwhile, circadian rhythm disturbances can affect the modulation of various physiological activities of human body. For example, they can lead to pathological deposition of *α*-synuclein in the locus coeruleus, brainstem reticular formation, dorsolateral tegmental nucleus, and pontine peduncle nucleus by inducing neuroinflammation, impaired protein homeostasis, and redox homeostasis. Their degeneration can cause the abnormal awakening-sleep transition, and then the phenomenon of RBD [27–29]. Both the gut microbiota and colonic motility have their circadian rhythms, and disruption of their circadian rhythms can also result in intestinal flora disturbances and colonic motility abnormalities, which in turn lead to gastrointestinal symptoms [30]. In addition, there is extensive functional overlap between the neural circuits that control thermoregulation in the body and the circadian system. Especially in the pons and medulla oblongata, circadian rhythm disturbances will induce abnormal temperature regulation such as fear of cold and heat [31].

The article "The Importance of Early Identification for Parkinson's Disease Patients with Postural Instability and Gait Disturbance" was retracted in 2023. Reasons: signs of a paper mill; compromised peer review; unreliable results or conclusions.

Although it was hard to judge completely whether there is an absolute causal relationship between RBD, gastrointestinal symptoms, thermoregulation dysfunction, and circadian rhythm disturbances through retrospective study, it was certain that the process of aging is accompanied by the disorder of biological clock and the circadian rhythm disturbances. Besides, sleep, defecation, and thermoregulation are all directly or indirectly modulated by circadian rhythms; thus, it can be said that circadian rhythm disturbances are important factors that cannot be ignored in the progression of PD. For the clinical treatment of PD, in addition to symptomatic treatment for the corresponding symptoms, modulating the circadian rhythms may also be one of the ways to achieve the overall regulation of PD, which have been verified by some clinical research results. For instance, bright light therapy (BLT), exogenous melatonin supplementation, deep brain stimulation, and other methods can not only improve the motor symptoms of PD, but also improve its RBD, gastrointestinal symptoms, excessive sweating, mood, and other nonmotor symptoms [30, 32–36]. As a result, pharmacological and nonpharmacological interventions targeting circadian rhythms may become a new strategy to delay the clinical progression of early PD.

The article "The Importance of Early Identification for Parkinson's Disease Patients with Postural Instability and Gait Disturbance" was retracted in 2023. Reasons: signs of a paper mill; compromised peer review; unreliable results or conclusions.

Over the past thirty years, a growing number of clinical studies have realized the importance of early identification and intervention of the subtypes of PD patients. However, before the development of Parkinson's disease, the symptoms of the clinical syndromes, such as constipation and insomnia, are so common that it is difficult to be the chief complaint for patients to seek medical treatment, or the main basis for doctors to diagnose diseases. In addition, the lack of typical motor symptoms also leads to the lack of criteria for efficacy evaluation. Thus, the transformation of different motor subtypes of PD in the clinical progress and the evolution of subtype-related influencing factors need to be further supported by multi-center, large-sample prospective investigations in the future so as to establish more intuitive criteria for syndrome diagnosis and the indicator architecture for evaluation of treatment efficacy. Moreover, the role of modulating circadian rhythms in improving clinical symptoms of PD also needs to be further verified by evidence-based medicine.

## 5. Conclusion

In conclusion, through this study, we found that the early identification of TD patients and PIGD patients is particularly important. NMS risk factors associated with PIGD were identified, including RBD, gastrointestinal symptoms, and thermoregulation. These findings may offer relevant basis for the development of individualized long-term management of PD subtypes in the future.

## Figures and Tables

**Figure 1:** Percentage of PD patients with H&Y stage 1 to 3 in different motor subtypes (abbreviations: TD, tremor-dominant; PIGD, postural instability and gait difficulty dominant; stage 1∼3, Hoehn and Yahr stage 1∼3).

**Figure 2:** Receiver operating characteristic (ROC) curve analysis of risk factors for PD-PIGD patients (abbreviations: RBDSQ, rapid eye movement sleep behavior disorder (RBD) screening questionnaire; PIGD, postural instability and gait difficulty dominant; UPDRS, Unified Parkinson's Disease Rating Scale; LED, levodopa equivalent dose). Larger area under the ROC curve indicates better prediction ability.

**Table 1:** Demographic factors of the TD and PIGD patients.

	TD (*n* = 148)	PIGD (*n* = 122)	*P*-value
*n* (male/female)	148 (83/65)	122 (67/55)	0.848
Age (years)	66.30 ± 8.75	66.55 ± 9.36	0.507
Education (years)	12.51 ± 2.83	11.67 ± 3.58	0.322
Age of onset(years)	62.03 ± 9.60	60.63 ± 10.25	0.127
PD family history			
No	137 (92.6)	112 (91.8)	0.846
Yes	11 (7.4)	10 (8.2)	
Disease duration (years)	4.28 ± 3.77	5.92 ± 4.57	0.001
Hoehn and Yahr stage	1.63 ± 0.53	2.00 ± 0.60	<0.001
LED (mg/day)	343.40 ± 199.63	486.13 ± 238.04	<0.001

The article "The Importance of Early Identification for Parkinson's Disease Patients with Postural Instability and Gait Disturbance" was retracted in 2023. Reasons: signs of a paper mill; compromised peer review; unreliable results or conclusions.

**Table 2:** Clinical characteristics of the TD and PIGD patients.

	TD (*n* = 148)	PIGD (*n* = 122)	*P*-value
UPDRS	21.53 ± 10.52	27.71 ± 11.09	<0.001
UPDRS Part I	2.1 ± 1.6	2.7 ± 2.0	0.007
UPDRS Part II	8.8 ± 4.8	11.3 ± 5.3	<0.001
UPDRS Part III	12.0 ± 6.0	13.7 ± 5.6	0.009
UPDRS Part IV	1.3 ± 1.6	1.6 ± 1.7	0.053
Tremor score	4.21 ± 1.67	1.22 ± 1.46	<0.001
PIGD score	2.24 ± 1.68	5.55 ± 2.76	<0.001
Rigidity score	0.80 ± 0.88	1.00 ± 1.06	0.057
Bradykinesia score	4.33 ± 2.52	5.53 ± 2.55	<0.001
SCOPA-AUT	6.80 ± 5.08	10.89 ± 7.15	<0.001
Gastrointestinal (Q1–7)	2.71 ± 2.37	4.29 ± 2.89	<0.001
Urinary (Q8–13)	2.48 ± 2.32	2.72 ± 3.08	0.056
Cardiovascular (Q14–16)	0.58 ± 0.93	0.83 ± 1.28	0.342
Thermoregulatory (Q17–21)	0.91 ± 1.49	1.91 ± 2.22	<0.001
Pupillomotor symptom (Q19)	0.07 ± 0.28	0.13 ± 0.48	0.460
Sexual (Q22–25)	0.05 ± 0.29	0.02 ± 0.18	0.256
PDSS	117.36 ± 20.44	114.05 ± 21.79	0.227
RBDSQ	1.46 ± 2.02	2.86 ± 2.35	<0.001
HAMA	8.23 ± 6.24	10.69 ± 6.99	0.003
Somatic anxiety	2.97 ± 2.67	4.33 ± 3.04	<0.001
Psychic anxiety	5.26 ± 4.09	6.36 ± 4.63	0.056
HAMD	31.39 ± 5.63	34.36 ± 7.38	<0.001

**Table 3:** Prevalence of nonmotor symptoms between TD and PIGD subtypes.

	The whole group	TD (*n* = 148)	PIGD (*n* = 122)	*P*-value
*Gastrointestinal symptoms*				
Dysphagia	54 (20.0)	14 (9.5)	40 (32.8)	<0.001
Sialorrhea	150 (55.6)	73 (49.3)	77 (63.1)	0.023
Abdominal fullness	51 (18.9)	21 (14.2)	30 (24.6)	0.030
Constipation	164 (60.7)	73 (49.3)	91 (74.6)	<0.001
Straining for defecation	180 (66.7)	89 (60.1)	91 (74.6)	0.012
Fecal incontinence	18 (6.7)	11 (7.4)	7 (5.7)	0.652

*Urinary symptoms*				
Pollakisuria	88 (32.6)	46 (31.1)	42 (34.4)	0.066
Nocturia	210 (77.8)	111 (75)	99 (81.1)	0.051

Cardiovascular symptoms				
Lightheaded (standing up)	81 (30.0)	45 (30.4)	36 (29.5)	0.843
Syncope	10 (3.7)	5 (3.4)	5 (4.1)	0.592

*Thermoregulatory symptoms*				
Hyperhidrosis (day)	83 (30.7)	34 (23)	49 (40.2)	0.002
Hyperhidrosis (night)	66 (24.4)	26 (17.6)	40 (32.8)	0.004
Cold intolerance	57 (21.1)	28 (18.9)	29 (23.8)	0.305
Heat intolerance	58 (21.5)	22 (14.9)	36 (29.5)	0.004

*Sleep disorders*				
Sleep onset insomnia	222 (82.2)	123 (83.1)	99 (81.1)	0.693
Sleep maintenance insomnia	229 (84.8)	128 (86.7)	101 (82.8)	0.385
Daytime sleepiness	198 (73.3)	108 (72.9)	90 (73.8)	0.874
RBD	55 (20.4)	17 (11.5)	38 (31.1)	<0.001

*Emotional disorders*				
Anxiety	163 (60.4)	79 (53.4)	84 (68.9)	0.010
Depression	231 (85.6)	112 (75.7)	119 (97.5)	<0.001

**Table 4:** Associations between each influence factor and disease severity in TD-PD patients.

Variables	TD			
	Univariable regression		Multivariable regression	
	OR (95% CI)	*P*-value	OR (95% CI)	*P*-value
Age (years)	1.024 (0.980–1.070)	0.285	—	—
Age of onset (years)	0.980 (0.950–1.011)	0.198	—	—
Disease duration (years)	1.364 (1.235–1.505)	<0.001	1.332 (1.194–1.486)	<0.001
LED (mg/day)	1.003 (1.002–1.005)	<0.001	1.002 (1.000–1.004)	0.011
Total UPDRS	1.098 (1.064–1.134)	<0.001	—	—
Tremor score	1.439 (1.125–1.842)	0.004	—	—
PIGD score	1.767 (1.453–2.148)	<0.001	1.207 (0.882–1.652)	0.039
Rigidity score	2.028 (1.427–2.883)	<0.001	—	—
Bradykinesia score	1.441 (1.265–1.643)	<0.001	—	—
Total SCOPA-AUT	1.149 (1.080–1.222)	<0.001	—	—
Gastrointestinal (Q1–7)	1.344 (1.178–1.534)	<0.001	—	—
Urinary (Q8–13)	1.364 (1.190–1.562)	<0.001	—	—
Cardiovascular (Q14–16)	1.219 (0.888–1.676)	0.220	—	—
Thermoregulatory (Q17–21)	0.962 (0.789–1.171)	0.697	—	—
Pupillomotor symptom (Q19)	2.475 (0.859–7.135)	0.093	—	—
Sexual (Q22–25)	0.592 (0.210–1.673)	0.323	—	—
RBDSQ	1.038 (0.897–1.201)	0.615	—	—
Total PDSS	0.990 (0.977–1.005)	0.203	—	—
Total HAMA	1.079 (1.028–1.133)	0.002	—	—
Total HAMD	1.069 (1.013–1.127)	0.014	—	—

The article "The Importance of Early Identification for Parkinson's Disease Patients with Postural Instability and Gait Disturbance" was retracted in 2023. Reasons: signs of a paper mill; compromised peer review; unreliable results or conclusions.

**Table 5:** Associations between each influence factor and disease severity in PIGD-PD patients.

Variables	PIGD				
	Univariable		Multivariable		
	OR (95% CI)	*P*-value	OR (95% CI)		*P*-value
Age (years)	0.995 (0.962–1.030)	0.777	—		—
Age of onset (years)	0.974 (0.943–1.005)	0.102	—		—
Disease duration (years)	1.138 (1.056–1.226)	0.001	—		—
LED (mg/day)	1.003 (1.001–1.004)	<0.001	—		—
Total UPDRS	1.126 (1.086–1.167)	<0.001	—		—
Tremor score	1.537 (1.097–2.155)	0.013	—		—
PIGD score	2.184 (1.766–2.701)	<0.001	1.922 (1.438–2.568)		<0.001
Rigidity score	1.875 (1.353–2.579)	<0.001	—		—
Bradykinesia score	1.302 (1.140–1.487)	<0.001	—		—
Total SCOPA-AUT	1.078 (1.029–1.129)	0.002	—		—
Gastrointestinal (Q1–7)	1.223 (1.089–1.372)	0.001	1.406 (1.073–1.841)		0.036
Urinary (Q8–13)	1.120 (1.008–1.245)	0.034	—		—
Cardiovascular (Q14–16)	1.223 (0.951–1.572)	0.117	—		—
Thermoregulatory (Q17–21)	1.146 (0.991–1.325)	0.065	—		—
Pupillomotor symptom (Q19)	1.936 (0.977–3.838)	0.058	—		—
Sexual (Q22–25)	1.871 (0.315–11.102)	0.490	—		—
RBDSQ	1.173 (1.021–1.347)	0.024	—		—
Total PDSS	1.007 (0.992–1.022)	0.346	—		—
Total HAMA	1.039 (0.992–1.087)	0.105	—		—
Total HAMD	1.052 (1.007–1.099)	0.023	—		—

**Table 6:** Regression analysis to identify risk factors for PIGD-PD subtype.

Variables	PIGD				
	Univariable		Multivariable		
	OR (95% CI)	*P*-value	OR (95% CI)	*P*-value	B
Age (years)	0.997 (0.968–1.028)	0.870	—	—	—
Age of onset (years)	0.986 (0.961–1.011)	0.260	—	—	—
Disease duration (years)	1.107 (1.041–1.178)	0.001	—	—	—
LED (mg/day)	1.003 (1.002–1.004)	<0.001	1.004 (1.001–1.007)	0.022	0.004
Total UPDRS	1.055 (1.030–1.081)	<0.001	1.198 (1.014–1.416)	0.034	0.181
Tremor score	0.208 (0.146–0.296)	<0.001	0.015 (0.003–0.066)	<0.001	-4.221
PIGD score	1.880 (1.593–2.219)	<0.001	4.116 (1.981–8.552)	<0.001	1.415
Rigidity score	1.369 (1.064–1.761)	0.015	—	—	—
Bradykinesia score	1.206 (1.092–1.331)	<0.001	—	—	—
Total SCOPA-AUT	1.124 (1.072–1.178)	<0.001	—	—	—
Gastrointestinal (Q1–7)	1.260 (1.140–1.393)	<0.001	1.808 (0.916–3.569)	0.048	0.592
Urinary (Q8–13)	1.193 (1.082–1.315)	<0.001	—	—	—
Cardiovascular (Q14–16)	1.227 (0.983–1.531)	0.070	—	—	—
Thermoregulatory (Q17–21)	1.342 (1.163–1.548)	<0.001	1.974 (0.932–4.182)	0.046	0.680
Pupillomotor symptom (Q19)	1.559 (0.807–3.012)	0.186	—	—	—
Sexual (Q22–25)	0.563 (0.176–1.803)	0.333	—	—	—
RBDSQ	1.332 (1.186–1.497)	<0.001	1.416 (1.053–1.903)	0.021	0.348
Total PDSS	0.993 (0.981–1.004)	0.200	—	—	—
Total HAMA	1.058 (1.019–1.099)	0.003	—	—	—
Total HAMD	1.075 (1.033–1.119)	<0.001	—	—	—

The article "The Importance of Early Identification for Parkinson's Disease Patients with Postural Instability and Gait Disturbance" was retracted in 2023. Reasons: signs of a paper mill; compromised peer review; unreliable results or conclusions.

**Table 7:** Regression analysis to identify risk factors for TD-PD subtype.

Variables	TD				
	Univariable		Multivariable		
	OR (95% CI)	*P*-value	OR (95% CI)	*P*-value	B
Age (years)	1.003 (0.973–1.033)	0.870	—	—	—
Age of onset (years)	1.015 (0.989–1.040)	0.260	—	—	—
Disease duration (years)	0.903 (0.849–0.961)	0.001	—	—	—
LED (mg/day)	0.997 (0.996–0.998)	<0.001	0.996 (0.993–0.999)	0.022	−0.004
Total UPDRS	0.948 (0.925–0.971)	<0.001	0.835 (0.706–0.986)	0.034	−0.181
Tremor score	4.812 (3.374–6.863)	<0.001	68.126 (15.124–306.862)	<0.001	4.221
PIGD score	0.532 (0.451–0.628)	<0.001	0.243 (0.117–0.505)	<0.001	−1.415
Rigidity score	0.730 (0.568–0.940)	0.015	—	—	—
Bradykinesia score	0.830 (0.751–0.916)	<0.001	—	—	—
Total SCOPA-AUT	0.890 (0.849–0.933)	<0.001	—	—	—
Gastrointestinal (Q1–7)	0.794 (0.718–0.878)	<0.001	0.553 (0.280–1.091)	0.048	−0.592
Urinary (Q8–13)	0.839 (0.760–0.925)	<0.001	—	—	—
Cardiovascular (Q14–16)	0.815 (0.653–1.017)	0.070	—	—	—
Thermoregulatory (Q17–21)	0.745 (0.646–0.860)	<0.001	0.506 (0.239–1.073)	0.046	−0.680
Pupillomotor symptom (Q19)	0.641 (0.332–1.239)	0.186	—	—	—
Sexual (Q22–25)	1.776 (0.555–5.688)	0.333	—	—	—
RBDSQ	0.751 (0.668–0.843)	<0.001	0.706 (0.526–0.949)	0.021	−0.348
Total PDSS	1.008 (0.996–1.019)	0.200	—	—	—
Total HAMA	0.945 (0.910–0.981)	0.003	—	—	—
Total HAMD	0.093 (0.894–0.968)	<0.001	—	—	—

**Table 8:** The results of the ROC analysis of risk factors of different motor subtypes.

Motor subtype	Variables	The optimum cut-off value	Sensitivity (%)	Specificity (%)	AUC	*P*-value
PIGD-PD	LED (mg/day)	331	74.4	56.5	0.681	<0.001
	Total UPDRS	26.5	52.1	70.7	0.662	<0.001
	PIGD score	3.5	66.9	77.6	0.802	<0.001
	Gastrointestinal	4.5	45.5	82.3	0.743	<0.001
	Thermoregulatory	1.5	50.4	73.5	0.665	<0.001
	RBDSQ	2.5	53.7	76.2	0.702	<0.001

TD-PD	Tremor score	1.5	80.3	89.9	0.892	<0.001

The article "The Importance of Early Identification for Parkinson's Disease Patients with Postural Instability and Gait Disturbance" was retracted in 2023. Reasons: signs of a paper mill; compromised peer review; unreliable results or conclusions.

## Data Availability

The data used to support the findings of this study are available from the corresponding author upon request.
